The article "hsa_circ_0084811 Regulates Cell Proliferation and Apoptosis in Retinoblastoma through miR-18a-5p/miR-18b-5p/E2F5 Axis" was retracted in 2024. Reasons: signs of a paper mill; suspected computer-generated content; unreliable results or conclusions; concerns about the data.

# hsa_circ_0084811 Regulates Cell Proliferation and Apoptosis in Retinoblastoma through miR-18a-5p/miR-18b-5p/E2F5 Axis

**DOI:** 10.1155/2022/6918396

**Published:** 2022-07-19

**Authors:** Guangwei Jiang, Mingxuan Qu, Lili Kong, Xiaoming Song, Shanhao Jiang

**Affiliations:** ^1^Department of Ophthalmology, Yantai Affiliated Hospital of Binzhou Medical University, Yantai City, Shandong Province 264100, China; ^2^Hemodialysis Room, Yantai Affiliated Hospital of Binzhou Medical University, Yantai City, Shandong Province 264100, China; ^3^Endocrinology & Metabolic Diseases, Yantai Affiliated Hospital of Binzhou Medical University, Yantai City, Shandong Province 264100, China

## Abstract

**Background:**

Retinoblastoma (RB) is the commonest primary intraocular malignancy during childhood. Circular RNAs (circRNAs) act as regulators in RB development, and hsa_circ_E2F5 (circ_0084811 in this study) was found to be highly expressed in RB cells, so we wanted to identify its detailed molecular mechanism.

**Methods:**

The expression level of circ_0084811 in RB cells was tested by RT-qPCR and its effects on RB cells were evaluated through functional assays. The regulatory mechanism that circ_0084811 may exert in RB progression was testified through mechanism experiments.

**Results:**

High circ_0084811 expression in RB cells facilitated cell proliferation but inhibited cell apoptosis. The enrichment of acetylation of histone 3 lysine 27 (H3K27ac) in circ_0084811 promoter induced circ_0084811 upregulation. Moreover, circ_0084811 regulated E2F transcription factor 5 (E2F5) expression via sponging microRNA-18a-5p (miR-18a-5p) and microRNA-18b-5p (miR-18b-5p).

**Conclusion:**

circ_0084811 modulated RB progression via the miR-18a-5p/miR-18b-5p/E2F5 axis.

## 1. Background

Retinoblastoma (RB) is defined as a malignant tumor which derives from the developing retina, and it accounts for 3% of all childhood cancers [1, 2]. The commonest signs of RB include white eye reflex and strabismus [3]. Although RB is a rare cancer among children, it is widely considered to be the most frequent primary intraocular malignancy during childhood [4]. According to statistics, the survival rate of RB patients has been improved a lot in developed countries but remains low in developing countries [5]. In this regard, exploring the development of RB from the perspective of molecular mechanism may be of great value to the treatment of RB [6].

Noncoding RNAs (ncRNAs) are defined as a heterogeneous class of RNAs which is limited in coding proteins. As a common type of ncRNAs, circular RNAs (circRNAs) are defined as covalently closed RNA molecules produced by back-splicing. Growing evidence has identified the great importance of circRNAs in tumors [7]. For instance, Liu et al. have proposed that hsa_circ_001783 accelerates the development of breast cancer through sequestering miR-200c-3p [8]. Lu et al. have proved that circSLC8A1 plays a suppressive role in bladder cancer via the crosstalk with the miR-130b/miR-494/PTEN axis [9]. Yu et al. have mentioned that circRNA_100876 exacerbates the proliferation and metastasis of gastric cancer via enhancing MIEN1 expression [10]. Moreover, circRNAs have been reported to participate in ocular diseases including RB [11]. For example, Jiang et al. have disclosed that circ_0000034 exacerbates the malignant development of RB through the miR-361-3p/ADAM19 axis [12]. Zhao et al. have uncovered that circ_0075804 boosts cell proliferation in RB through recruiting HNRNPK protein and stabilizing E2F3 mRNA [13]. Xing et al. have implied that hsa_circ_0001649 modulates RB malignancy through modulation of the AKT/mTOR signaling pathway [14].

The E2F family of transcription factors has been illustrated as a key regulator related to the proliferation, differentiation, and apoptosis of a variety of tissues [15]. E2F transcription factor 5 (E2F5), a member of E2F family, has been characterized as a transcriptional repressor which can regulate cell proliferation through its interaction with the RB protein for inhibition of target gene transcription. In addition, it has been documented to play critical roles in cancer development, including RB [16, 17]. Since circRNAs can be transcribed together with their parental genes and, in turn, they can regulate the transcription of the parental gene or related genes [18], we explored whether circ_0084811 may regulate its host gene E2F5 in RB.

## 2. Methods

### 2.1. Cell Culture

RB cells (HXO-Rb44, Y79, SO-Rb50, and WERI-Rb-1) and human retinal pigment epithelial ARPE-19 cell line were selected for this study. Y79, WERI-Rb-1, and ARPE-19 cells were bought from ATCC (Manassas, VA, USA). HXO-Rb44 cell line was obtained from Zishi Biotechnology Co., Ltd. (Shanghai, China) while SO-Rb50 cell line was bought from Huatuo Biotechnology Co., Ltd. (Shenzhen, China). The four RB cell lines were cultivated in RPMI-1640 medium while ARPE-19 cell line was cultured in DMEM: F12 medium. All the above mediums were treated with 10% FBS in humidified air, with the culture condition set as 37°C, 5% CO_2_.

### 2.2. Cell Transfection

The shRNAs targeting CBP (sh-CBP#1/2), circ_0084811 (sh-circ_0084811#1/2/3), or E2F5 (sh-E2F5#1/2) were designed and synthesized by RiboBio (Guangzhou, China). For the overexpression of E2F5, the sequence was subcloned into pcDNA 3.1 vectors with empty pcDNA3.1 vector as the negative control. Besides, miR-18a-5p mimics/inhibitor, miR-18b-5p mimics/inhibitor, and their respective negative controls (control mimics/NC inhibitor) were also constructed by RiboBio. Transfection was performed by using Lipofectamine 3000 (Invitrogen) for 48 h.

### 2.3. Total RNA Extraction and Quantitative Real-Time Polymerase Chain Reaction (RT-qPCR) Analysis

In line with the instruction of TRIzol reagent (Invitrogen), the isolation of total RNA samples was extracted in RB cells. RNA concentration was detected by NanoDrop 2000 (Thermo Scientific, USA). Synthesis of complementary DNA (cDNA) was carried out using the PrimeScript™ RT master mix (Takara, Japan). RT-qPCR reaction was achieved with SYBR Green PCR Master Mix (Applied Biosystems) followed by the 2^-*ΔΔ*CT^ method. GAPDH and U6 were used as internal controls. The experimental procedure was independently carried out in triplicate. Detailed sequences are provided in Supplementary Table 1.

### 2.4. MTT Assay

Transfected cells were seeded in 96-well plates (200 *μ*L, 3 × 10^3^ cells/well) added with 10 *μ*L MTT (5 mg/mL) in each well. After incubation for 4 h, the precipitates were dissolved in dimethyl sulfoxide (DMSO, 100 *μ*L). The absorbance was measured at 490 nm under a microplate spectrophotometer. Experiments were independently carried out in triplicate.

### 2.5. Soft Agar Assay

After transfection, RB cells were plated in 6-well plates. After 2-4 weeks, cells were maintained in an upper layer of 0.35% agarose (Lonza Rockland) in DMEM added with 10% FBS. With the utilization of 0.5% basal agar and 10% FBS, suspend cells were overlaid and kept under room temperature until the solidification of agarose. Finally, images of cell colonies were taken. The experiment went through three independent repeats.

### 2.6. Subcellular Fractionation

PARIS™ Kit (Ambion, Austin, TX) was used to separate cytoplasmic and nuclear elements in accordance with the user guide. Cell cytoplasm was isolated by adding the cell fractionation buffer, and cell disruption buffer was used to collect cell nucleus. GAPDH was the cytoplasmic control and U6 was the nuclear control. The assay went through three independent repeats.

### 2.7. Fluorescent In Situ Hybridization (FISH) Assay

The circ_0084811-specific RNA FISH probe (CTGAAGATATCACCTGTAAG-biotin) was procured from RiboBio for cellular analysis according to the instruction of the provider. The fixed cell samples were rinsed in PBS and then dehydrated. After that, the air-dried cells were hybridized with FISH probe in hybridization buffer and then treated with DAPI staining reagent. Nuclei were counterstained with DAPI, and finally, an Olympus fluorescent microscope was applied for image observation. The assay went through three independent repeats.

### 2.8. RNA Pull-Down Assay

RB cells were treated with a biotinylated circ_0084811 probe. Magnetic beads were then added into cells. The precipitated product collected by beads was purified for RT-qPCR analysis. The biotin-labeled circ_0084811 probe with Bio-NC was designed and synthesized by RiboBio (Guangzhou, Guangdong, China). Cells were lysed with lysis buffer, and then, the lysates were incubated with specific biotin-labeled probes for 2 h. Then, the mixtures were incubated with the streptavidin beads to pull down the biotin-labeled RNA complex for another 4 h. After washing, the RNA complex was extracted with TRIzol and the enrichment of miR-654-3p, miR-18b-5p, and miR-18a-5p was examined via RT-qPCR assay. The experiment was subject to three independent repeats.

### 2.9. RNA Immunoprecipitation (RIP) Assay

In accordance with the user guide, Magna RIP RNA-Binding Protein Immunoprecipitation Kit (Millipore, Bedford, MA) was used for RIP assay. Cells were lysed with RNA lysis buffer, and then, Ago2 antibody (Abcam, ab186733; 1/30-1/50) and IgG antibody (Abcam, ab172730; 1-2 *μ*g/mL) were used to immunoprecipitate cell lysates. Finally, the RNA complexes were extracted for RT-qPCR analysis. The experiment was subject to three independent repeats.

### 2.10. Chromatin Immunoprecipitation (ChIP) Assay

ChIP assay was implemented utilizing ChIP Assay Kit (Beyotime, Shanghai, China). In short, BC cell lysates were sonicated to be fragments and immunoprecipitated using anti-H3K27AC (BioVision, 6869-25, 1-2 *μ*L) or anti-CBP (Abcam, ab154532; 1/500-1/3000) with immunoglobulin G (IgG) antibody (Abcam; ab172730; 1-2 *μ*g/mL) as a negative control. The immunoprecipitated DNA was extracted for RT-qPCR analysis. The experiment went through three independent repeats.

### 2.11. Luciferase Reporter Assay

The fragments of circ_0084811 or E2F5 mRNA covering wild-type (Wt) and mutant-type (Mut) miR-18a-5p or miR-18b-5p binding sites were inserted into pmirGLO dual-luciferase vector to construct pmirGLO-circ_0084811-Wt/Mut and pmirGLO-E2F5 3′UTR-Wt/Mut, respectively. Later, the reporter gene went through the cotransfection with control mimics and miR-18a-5p or miR-18b-5p mimics into RB cells for 48 h. Dual-luciferase reporter assay system (Promega) was eventually applied to measure the luciferase activity. The assay was subject to three independent repeats.

### 2.12. Western Blot Assay

Total cell lysates were extracted using RIPA lysis buffer (Thermo Fisher, USA), followed by using a BCA protein assay reagent (Beyotime) to confirm the protein concentration. After being separated through SDS-PAGE (sodium dodecyl sulfate polyacrylamide gel electrophoresis), proteins were transferred to polyvinylidene fluoride (PVDF) membranes and cultured in 5% skim milk. The membrane was incubated with the primary antibodies, including CBP (ab119488, Abcam; 1/500-1/3000), BCL2 (ab196495, Abcam; 1/1000), Bax (ab32503, Abcam; 1/1000-1/10000), Cleaved caspase-3 (ab2302, Abcam; 1/500), total caspase-3 (EPX01A-12012-901, Thermo Fisher; 1/5000), E2F5 (ab59769, Abcam; 1/5000-1/20000), *β*-actin (ab6276, Abcam; 1/5000-1/16000), and GAPDH (ab8245, Abcam; 1/500-1/10000) overnight at 4°C. Subsequently, the membranes were incubated with horseradish peroxidase-labeled secondary antibodies. By using Clarity Max Western ECL Substrate (Bio-Rad), we confirmed the protein bands. The experiment was subject to three independent repeats.

### 2.13. Statistical Analysis

All the experiments went through three independent repeats. The analysis of data was conducted by SPSS 22.0 statistical software package. All data were exhibited as mean ± standard deviation (SD). The group differences between two or more groups were analyzed using Student's *t*-test or one-way ANOVA. The significance of statistics was set at *P* < 0.05 (∗) or *P* < 0.01 (∗∗).

## 3. Results

### 3.1. circ_0084811 Was Highly Expressed in RB Cells, and Its Loop Structure Was Confirmed

As we have illustrated before, we have known that E2F5 is associated with RB, and we wanted to find the potential circRNA which was cyclized from E2F5 and their interaction in RB, so we performed experiments with the aim to verify the target circRNA whose host gene is E2F5 in RB cells and to further verify their regulatory mechanism. Through the circBank database (http://www.circbank.cn/index.html), we found four circRNAs whose gene symbol was E2F5, which were hsa_circ_E2F5_001 (circBase_id: circ_0084811), hsa_circ_E2F5_002 (circBase_id: circ_0137212), hsa_circ_E2F5_003 (circBase_id: circ_0137213), and hsa_circ_E2F5_004 (circBase_id: circ_0137214) (Figure 1(a), left). Then, we examined their expression in RB cell lines (HXO-Rb44, Y79, SO-Rb50, and WERI-Rb-1) and normal ARPE-19 cell line and found that only circ_0084811 was with obviously high expression in RB cell lines (Figure 1(a), right). The schematic diagram of the genomic location of circ_0084811 is demonstrated in Figure 1(b). After RNase R treatment, linear-E2F5 level was observably reduced while circ_0084811 level had no variation, which verified the loop structure of circ_0084811 (Figure 1(c)). The specific convergent and divergent primers were, respectively, designed to amplify the linear and back-splicing forms of E2F5, and circ_0084811 was only amplified by cDNA templates instead of genomic DNA (gDNA) templates (Figure 1(d)). After adding actinomycin D (Act D), circ_0084811 displayed a longer half-life in comparison with linear E2F5, indicating its stable form (Figure 1(e)).

### 3.2. H3K27ac Activated circ_0084811 Expression in RB Cells

Increasing studies have elaborated the critical role of histone acetylation in gene expression [19]. Moreover, many reports have illustrated that RNAs are upregulated by H3K27ac modification at promoter region to transcriptionally activate the expression of these RNAs, which suggests the crucial role of H3K27ac in cancer progression [20–23]. Therefore, we wanted to explore the H3K27ac level in the promoter region of circ_0084811. According to the search results of UCSC (http://genome.ucsc.edu/), H3K27ac was enriched in the promoter of circ_0084811 (Figure 2(a)). The result of ChIP assay also suggested that H3K27ac was highly enriched in the promoter region of circ_0084811 in RB cells (Figure 2(b)). Additionally, we observed that after the treatment of C646, the histone acetyltransferase inhibitor, circ_0084811 expression decreased (Figure 2(c)). CBP is a crucial factor in chromatin acetylation, so we made a conjecture that CBP might also contribute to the acetylation. CBP was tested to be with high expression in RB cells (Figure 2(d)), and circ_0084811 expression was reduced after sh-CRP#1/2 transfection was made in RB cells (Figures 2(e)–2(g)). Next, the considerable enrichment of CBP in the circ_0084811 promoter showed the binding ability between them, as exhibited by ChIP assay (Figure 2(h)). We found that CBP deficiency impeded the binding between circ_0084811 promoter and H3K27ac (Figure 2(i)). In a word, the upregulation of circ_0084811 in RB cells was mediated by H3K27ac acetylation.

### 3.3. circ_0084811 Knockdown Hampered the Proliferation and Induced the Apoptosis of RB Cells

We tried to evaluate the impact circ_0084811 may exert on RB progression through a series of functional assays. First of all, we transfected sh-circ_0084811#1/2/3 in RB cells, and a favorable interference efficiency was observed (Figure 3(a)). It was confirmed from MTT assay and soft agar assay that cell viability as well as proliferation was declined by circ_0084811 depletion (Figures 3(b) and 3(c)). Moreover, the protein levels of apoptosis-related factors (BCL2, Bax, and Cleaved caspase-3) were confirmed via western blot, and results suggested that circ_0084811 downregulation decreased BCL2 protein level while Bax along with Cleaved caspase-3 displayed increased protein expression (Figure 3(d)). Overall, circ_0084811 promoted cell proliferation while it inhibited cell apoptosis in RB.

### 3.4. circ_0084811 Modulated E2F5 Expression

According to subcellular fractionation detection as well as FISH assay, the majority of circ_0084811 was in the cytoplasm of transfected cells (Figures 4(a) and 4(b)). It was then verified that E2F5 expression and protein level were lessened upon circ_0084811 silencing (Figures 4(c) and 4(d)). In view of the fact that E2F5 functions as a common transcription factor, we conducted RT-qPCR assay to verify whether E2F5 may influence the expression of circ_0084811. The expression of E2F5 was firstly knocked down by the transfection of sh-E2F5#1/2 plasmids, and then, we found that circ_0084811 expression was not influenced by E2F5 (Figures 4(e) and 4(f)). To conclude, E2F5 was positively regulated by circ_0084811 while E2F5 could not regulate the expression of circ_0084811.

### 3.5. circ_0084811 Sponged miR-18a-5p and miR-18b-5p to Regulate E2F5 Expression

With the application of starBase (http://starbase.sysu.edu.cn/), we could see that there were 3 potential miRNAs (miR-654-3p, miR-18b-5p, and miR-18a-5p) which had binding possibility to circ_0084811 and E2F5 (Figure 5(a)). We found through RNA pull-down assay that miR-18a-5p and miR-18b-5p were dramatically accumulated in the biotin-labeled circ_0084811 probe while no change could be seen in the miR-654-3p group (Figure 5(b)).  Figure 5(c) exhibited related binding sequences between these RNAs. After that, RIP assay was carried out, and it was observed that circ_0084811, miR-18a-5p, miR-18b-5p, and E2F5 were all enriched in Ago2 antibody rather than IgG antibody (Figure 5(d)). The expression of these two miRNAs was elevated in RB cells, and it was then observed that after their overexpression, the wild type of the circ_0084811 group and E2F5 3′UTR group both exhibited declined luciferase activity, while the according mutant groups were barely affected (Figures 5(e) and 5(f)). After that, miR-18a-5p and miR-18b-5p expression was reduced in RB cells (Figure 5(g)), and then, the expression of E2F5 in different transfection groups was analyzed. As shown by the results, decreased E2F5 expression after circ_0084811 silencing was partially restored by miR-18a-5p inhibitor or miR-18b-5p inhibitor (Figures 5(h) and 5(i)). Taken together, circ_0084811 targeted E2F5 via sequestering miR-18a-5p and miR-18b-5p.

### 3.6. circ_0084811 Promoted RB Progression via Modulating the miR-18a-5p/miR-18b-5p/E2F5 Axis

E2F5 was overexpressed in Y79 cells via using the pcDNA3.1/E2F5 vector for later rescue experiments (Figure 6(a)). At first, we found through MTT assay that circ_0084811 downregulation inhibited cell viability, but this impact was partially counteracted by the treatment of miR-18a-5p inhibitor or miR-18b-5p inhibitor, while E2F5 overexpression could fully reverse this effect (Figure 6(b)). The similar result was also seen in the soft agar assay (Figure 6(c)), which indicated that RB cell proliferation upon circ_0084811 silencing was regulated by the miR-18a-5p/miR-18b-5p/E2F5 axis. Subsequently, we adopted RT-qPCR as well as western blot assays to analyze RB cell apoptosis under different conditions, and it was shown that the declined BCL2 expression and protein levels caused by circ_0084811 silencing was partially counteracted by miR-18a-5p inhibition or miR-18b-5p inhibition while it was greatly recovered by E2F5 overexpression. Besides, the expression and protein levels of Bax and Cleaved caspase-3 showed opposite results (Figure 6(d)). The above results indicated that promoted cell apoptosis induced by circ_0084811 deficiency could be partially countervailed by the knockdown of miR-18a-5p or miR-18b-5p while it could be greatly counteracted by E2F5 upregulation. To sum up, the circ_0084811/miR-18a-5p/miR-18b-5p/E2F5 axis contributed to the progression of RB.

## 4. Discussion

In recent years, the significance of circRNAs in RB has been highlighted [24]. E2F5 has been commonly considered to act as an oncogene in cancers, which include prostate cancer, non-small-cell lung cancer, and ovarian cancer [25–27]. Moreover, it has been confirmed that E2F5 can boost RB progression by affecting cell proliferation, invasion, and tumor formation [17]. More importantly, it has been reported that some circRNAs can be transcribed together with their parental genes and in turn regulate the transcription of the parental gene or related genes [18], so we speculated that circRNAs which were cyclized from E2F5 might also exert certain impact on RB progression. In our study, circ_0084811 was discovered to be distinctly overexpressed in RB cells, and it was verified through mechanism experiments that the upregulation of circ_0084811 in RB cells was induced by the enrichment of H3K27ac in the circ_0084811 promoter. Functionally, inhibition of circ_0084811 diminished RB cell proliferation and stimulated cell apoptosis.

circRNAs functioning as miRNA sponges to influence mRNA translation or stability, thereby participating in the cellular activities in human cancers, have been widely documented [28]. Through our investigation, the cytoplasmic distribution of circ_0084811 in RB cells was identified, and we discovered that circ_0084811 also positively regulated the expression of E2F5. Hence, we speculated that circ_0084811 might sequester certain miRNAs to modulate E2F5 expression. With the application of the starBase database, 3 potential miRNAs were predicted. At the same time, miR-18a-5p and miR-18b-5p were selected to be the downstream target genes, which contributed to the malignant progression of RB. miR-18a-5p has been proven to inhibit the malignancy of ovarian cancer and hepatocellular carcinoma [29, 30]. Besides, miR-18b-5p has been demonstrated to repress lung adenocarcinoma, ovarian cancer, and liver cancer [31–33]. Through our investigations, we revealed the interaction of circ_0084811, miR-18b-5p, and E2F5 in RB and demonstrated that circ_0084811 had the further value to be studied as a competing endogenous RNA (ceRNA). Circular RNAs (circRNAs) sponging miRNAs (microRNAs) to further regulate the downstream gene expression have been well-elucidated by many researches [34]. In RB, the ceRNA model of circRNA_100782 sponging miR-574-3p to further modulate Rb expression is confirmed [35] and circ-E2F3 sponges miR-204-5p and positively regulates ROCK1 expression to promote cancer progression [36]. circ_0000527 functioning as a ceRNA to directly target miR-646 and positively regulate LRP6 expression in RB cells has also been elucidated [37]. What we have demonstrated about the ceRNA network in RB cells may help to enrich the current exploration of this regulatory mechanism in the regulation of RB malignancy.

## 5. Conclusion

All in all, circ_0084811 was demonstrated to be mediated by H3K27ac acetylation, and high circ_0084811 expression in RB cells hindered the malignant cell behaviors in RB. Furthermore, circ_0084811 aggravated the progression of RB through the miR-18a-5p/miR-18b-5p/E2F5 axis. Lack of clinical investigation is a main limitation of the current study. We will collect clinical samples to elaborate the clinical significance of the circ_0084811/miR-18a-5p/miR-18b-5p/E2F5 axis in RB in our future study.

## Figures and Tables

**Figure 1:** circ_0084811 was highly expressed in RB cells, and its loop structure was confirmed. (a) Potential circRNAs whose gene symbol was E2F5 were selected via the circBank database. Their expression in RB cell lines and normal cell line was tested via RT-qPCR. (b) The schematic diagram of the genomic location of circ_0084811. (c) circ_0084811 and linear E2F5 expression in RB cells treated with RNase R. (d) The loop structure of circ_0084811 confirmed through gel electrophoresis. (e) Relative RNA level of circ_0084811 and linear-E2F5 in RB cells treated with actinomycin D. Each assay went through three biological replicates. The sample number (*n*) = 3. ^∗^*P* < 0.05 and ^∗∗^*P* < 0.01.

**Figure 2:** H3K27ac activated the expression of circ_0084811 in RB cells. (a) H3K27ac level in the circ_0084811 promoter region was measured through the UCSC database. (b) The interaction between H3K27ac and the circ_0084811 promoter in RB cells was confirmed through ChIP analysis. (c) circ_0084811 expression in cells treated with C646. (d) CBP expression in RB cell lines and normal cell line. (e, f) CBP expression and protein level were decreased by sh-CBP transfection. (g) circ_0084811 expression was measured after CBP was silenced. (h) The binding ability between circ_0084811 promoter and CBP in RB cells was verified by ChIP assay. (i) The enrichment of circ_0084811 promoter in H3K27ac antibody when CBP was downregulated. Each assay went through three biological replicates. The sample number (*n*) = 3. ^∗∗^*P* < 0.01.

**Figure 3:** circ_0084811 knockdown hampered the proliferation and induced the apoptosis of RB cells. (a) circ_0084811 expression was decreased in RB cells by sh-circ_0084811 transfection. (b, c) MTT assay, together with soft agar assay (scale bar: 200 *μ*m), was conducted to observe cell proliferation upon circ_0084811 knockdown in RB. (d) The protein levels of apoptosis-related factors after circ_0084811 was depleted. Each assay went through three biological replicates. The sample number (*n*) = 3. ^∗∗^*P* < 0.01.

**Figure 4:** circ_0084811 modulated E2F5 expression. (a, b) The location of circ_0084811 in RB cells determined by subcellular fractionation along with FISH assay (scale bar: 10 *μ*m). (c, d E2F5 expression as well as protein level after circ_0084811 was silenced. (e) E2F5 expression was cut down in RB cells by the sh-E2F5 transfection. (f) circ_0084811 expression was tested when E2F5 was downregulated. Each assay went through three biological replicates. The sample number (*n*) = 3. ^∗∗^*P* < 0.01.

**Figure 5:** circ_0084811 sponged miR-18a-5p and miR-18b-5p to regulate E2F5 expression. (a) Potential miRNAs of circ_0084811 and E2F5 forecasted through starBase. (b) miR-654-3p, miR-18a-5p ,and miR-18b-5p enrichment in bio-circ_0084811 probe was confirmed via RNA pull-down assay. (c) Predicted binding sites between circ_0084811 and miR-18a-5p or miR-18b-5p, E2F5, and miR-18a-5p or miR-18b-5p. (d) The relationship among circ_0084811, miR-18a-5p, miR-18b-5p, and E2F5 was confirmed through RIP assay. (e) miR-18a-5p mimics and miR-18b-5p mimics were utilized to elevate their expression in RB cells. (f) The affinity of miR-18a-5p or miR-18b-5p with circ_0084811 or E2F5 was testified by luciferase reporter assays. (g) miR-18a-5p and miR-18b-5p were, respectively, silenced in RB cells by inhibitor transfection. (h, i) E2F5 expression in RB cells transfected with sh-NC, sh-circ_0084811#1, sh-circ_0084811#1+miR-18a-5p inhibitor, and sh-circ_0084811#1+miR-18b-5p inhibitor plasmids. Each assay went through three biological replicates. The sample number (*n*) = 3. ^∗^*P* < 0.05 and ^∗∗^*P* < 0.01.

**Figure 6:** circ_0084811 promoted RB progression via the miR-18a-5p/miR-18b-5p/E2F5 axis. (a) E2F5 expression in pcDNA3.1/E2F5-transfected cells. (b–d) The proliferative capacity of Y79 cells (b, c) as well as cell apoptosis in RB (d) was assessed in different transfection groups (scale bar for soft agar assay: 200 *μ*m). Each assay went through three biological replicates. The sample number (*n*) = 3. ^∗^*P* < 0.05 and ^∗∗^*P* < 0.01.

## Data Availability

The data used to support the findings of this study are included within the article.

## Abbreviations

RB: Retinoblastoma
circRNAs: Circular RNAs
E2F5: E2F transcription factor 5
miR-18a-5p: MicroRNA-18a-5p
miR-18b-5p: MicroRNA-18b-5p
ncRNAs: Noncoding RNAs
ceRNA: Competing endogenous RNA
ATCC: American Type Culture Collection
RT-qPCR: Quantitative reverse transcription real-time polymerase chain reaction
FISH: Fluorescent in situ hybridization
RIP: RNA immunoprecipitation
ChIP: Chromatin immunoprecipitation
IgG: Immunoglobulin G
Wt: Wild type
Mut: Mutant type
SD: Standard deviation
gDNA: Genomic DNA
Act D: Actinomycin D.

## Supplementary Materials

Supplementary Materials Supplementary Table 1: related sequences utilized in this study.
